# Arginine methylation of SHANK2 by PRMT7 promotes human breast cancer metastasis through activating endosomal FAK signalling

This article has been retracted.

**DOI:** 10.7554/eLife.57617

**Published:** 2020-08-26

**Authors:** Yingqi Liu, Lingling Li, Xiaoqing Liu, Yibo Wang, Lingxia Liu, Lu Peng, Jiayuan Liu, Lian Zhang, Guannan Wang, Hongyuan Li, Dong-Xu Liu, Baiqu Huang, Jun Lu, Yu Zhang

**Affiliations:** 1 The Key Laboratory of Molecular Epigenetics of the Ministry of Education, Northeast Normal UniversityChangchunChina; 2 The Institute of Genetics and Cytology, Northeast Normal UniversityChangchunChina; 3 Laboratory of Chemical Biology, Changchun Institute of Applied Chemistry, Chinese Academy of SciencesChangchunChina; 4 The Centre for Biomedical and Chemical Sciences, School of Science, Faculty of Health and Environmental Sciences, Auckland University of TechnologyAucklandNew Zealand; University of AlbertaCanada; Memorial Sloan Kettering Cancer CenterUnited States

**Keywords:** metastasis, endocytosis, methylation, PRMT7, SHANK2, FAK, Human

## Abstract

Arginine methyltransferase PRMT7 is associated with human breast cancer metastasis. Endosomal FAK signalling is critical for cancer cell migration. Here we identified the pivotal roles of PRMT7 in promoting endosomal FAK signalling activation during breast cancer metastasis. PRMT7 exerted its functions through binding to scaffold protein SHANK2 and catalyzing di-methylation of SHANK2 at R240. SHANK2 R240 methylation exposed ANK domain by disrupting its SPN-ANK domain blockade, promoting in co-accumulation of dynamin2, talin, FAK, cortactin with SHANK2 on endosomes. In addition, SHANK2 R240 methylation activated endosomal FAK/cortactin signals in vitro and in vivo. Consistently, all the levels of PRMT7, methylated SHANK2, FAK Y397 phosphorylation and cortactin Y421 phosphorylation were correlated with aggressive clinical breast cancer tissues. These findings characterize the PRMT7-dependent SHANK2 methylation as a key player in mediating endosomal FAK signals activation, also point to the value of SHANK2 R240 methylation as a target for breast cancer metastasis.

## Introduction

Protein arginine methyltransferases (PRMTs) catalyze mono-methylation and symmetric or asymmetric di-methylation of arginine residues on both histone and non-histone substrates to modulate diverse biological processes, including transcription, cell signalling, mRNA translation, DNA damage repair signalling, receptor trafficking, protein stability and pre-mRNA splicing (Jelinic et al., 2006; Bedford and Clarke, 2009; Dhar et al., 2012; Jeong et al., 2016; Blanc and Richard, 2017; Jeong et al., 2020). Protein Arginine Methyltransferase 7 (PRMT7) was reported as a type III PRMT to catalyze mono-methylation of arginine residues on both histone and non-histone substrates (Bedford and Clarke, 2009; Karkhanis et al., 2012; Blanc and Richard, 2017; Jain and Clarke, 2019; Haghandish et al., 2019). Recent studies also reported that PRMT7 can symmetrically di-methylate proteins such as p38 and GLI2 (Jeong et al., 2020; Vuong et al., 2020). Others and our previous studies have linked PRMT7 to breast cancer progression. Specifically, our previous work reported that PRMT7 promoted metastasis of breast carcinoma cells by triggering EMT (epithelial-mesenchymal transition) program (Yao et al., 2014). PRMT7 can also upregulate the expression of matrix metalloproteinase nine to promote metastasis of breast cancer (Baldwin et al., 2015). We also found that PRMT7 was automethylated at residue R531, which potentiated the PRMT7-induced EMT program and metastasis (Geng et al., 2017).

Endocytosis of migrating cells is a fundamental process which is required for adhesion formation and efficient cell movement (Kaksonen and Roux, 2018; Scita and Di Fiore, 2010). Increasing evidence indicates that deregulated endocytosis is a relapse mechanism that contributes to the acquisition of malignant characteristics in tumour cells, including enhanced cell migration, invasion and metastasis (Hamidi and Ivaska, 2018; McMahon and Boucrot, 2011). During invasive cell migration, receptors are internalized through the cyclic trafficking of endosome and transported to early endosome before recycling back to the plasma membrane, consequently the cytoskeleton is polarized by actin polymerization via scaffold proteins, and forming a leading protrusion (Trusolino et al., 2010; Wang et al., 2011; Verma et al., 2015; Hamidi and Ivaska, 2018). The focal adhesion kinase (FAK) is a cytoplasmic protein-tyrosine kinase and plays a pivotal role in many cellular processes such as cell adhesion, survival and migration (Murphy and Courtneidge, 2011; Alanko and Ivaska, 2016; Schoenherr et al., 2018). During endocytosis, integrin or talin engages with FAK to co-localize on endosome. FAK undergos autophosphorylation on Y397, which results in cell dissemination (Alanko et al., 2015; Nader et al., 2016; Xiuping et al., 2018; Hamidi and Ivaska, 2018). Additionally, Y397 phosphorylation of FAK facilitates the association of FAK with actin-binding protein cortactin, which renders cortactin function in formation of lamellipodia and filopodia (Tomar et al., 2012; Eke et al., 2012; Wang et al., 2011). Although increased endosome recycling to the plasma membrane contributes to enhanced cell migration, the mechanism of endosomal assembly and signals activation is largely unknown. Recent reports also uncovered the connection between arginine methylation and phosphorylation with endocytic trafficking (Albrecht et al., 2018). However, whether PRMT7 promotes breast cancer metastasis through regulating endocytic traffic remains unclear.

Scaffolding proteins SH3 and multiple ankyrin repeat domains 2 (SHANK2) localizes in cytoplasm and plays important roles in regulating synapse plasticity (Lee et al., 2010; Naisbitt et al., 1999; Sala et al., 2001; Sheng and Kim, 2000; Tu et al., 1999). The SHANK family of master scaffolding proteins include three members, that is SHANK1, 2 and 3. SHANK family proteins have been linked to Autistic Spectrum Disorder (Lim et al., 1999; Mei et al., 2016; Monteiro and Feng, 2017; Yoon et al., 2017). Mutations in genes encoding SHANK family proteins (SHANK1, 2 and 3) often result in marked behavioural phenotypes in mice (Mameza et al., 2013; Schmeisser et al., 2012; Won et al., 2012), such as an increase in repetitive routines, altered social behaviour and anxiety-like phenotypes. Recent studies also linked SHANK family proteins to cancer cell invasion. SHANK1 and SHANK3 were reported to inhibit cell spreading, migration and invasion in cancer cells through sequestering active Rap1 and R-Ras (Lilja et al., 2017). However, the precise roles of SHANK2 in tumour progression have not been investigated.

In this study, we identified that SHANK2 was a new substrate of PRMT7. Methylation of SHANK2 at R240 by PRMT7 exposed ANK domain by disrupting its SPN-ANK domain blockade. Further, SHANK2 R240 methylation reinforced breast cancer cell migration through activating endosome FAK signalling. Collectively, these findings represent one mechanistic explanation for how PRMT7 regulating breast cancer cell metastasis by mediating endosome formation, and may provide potential clues for tumour metastasis treatment strategies.

## Results

### SHANK2 interacts with PRMT7 and is a substrate for PRMT7-mediated arginine methylation

To explore the mechanism of PRMT7 action in tumour metastatic progression, we used the Flag-tagged PRMT7 fusion protein as bait in mass spectrometry to pick up the possible regulatory factors, which might be directly regulated by PRMT7 (Figure 1A). The results revealed that PRMT7 is associated with multiple proteins including SHANK2, MRPS23, Plectin1, SNRPB and ARHGAP32. Among the PRMT7-interacting proteins, we chose SHANK2 as a target for a more detailed study. Although SHANK1 and SHANK3 have been reported to inhibit cancer cell migration (Lilja et al., 2017), whether SHANK2 plays a role in cancer progression is unknown. To determine whether PRMT7 methylates SHANK2, we first conducted a CoIP assay to confirm the binding between PRMT7 and SHANK2 (Figure 1B and C). We then incubated the purified GST-tagged PRMT7 with SHANK2 protein, and the results showed that they could interact with each other (Figure 1D). To map the SHANK2 regions that bind PRMT7, we expressed a series of truncated GST- SHANK2 (Figure 1E), and found that the SHANK2 ANK, PDZ and SAM domains were responsible for the interaction between PRMT7 and SHANK2 (Figure 1F). The interaction between PRMT7 and SHANK2 indicated that SHANK2 might be a new substrate of PRMT7.

**Figure 1.** PRMT7 methylated SHANK2. Immunoprecipitation and immunoblotting analyzes were performed with the indicated antibodies. (**A**) PRMT7 associated proteins from MCF7 cells expressing stable FLAG-PRMT7 were immunopurified with anti-FLAG (α-FLAG) affinity resins. The protein bands were analyzed by mass spectrometry. Representative peptide fragments of PRMT7 associated proteins and peptide coverage of the indicated proteins are shown. (**B**) HEK293T cells were co-transfected with Flag-PRMT7 and/or HA-SHANK2 plasmids. (**C**) Endogenous SHANK2 or PRMT7 was IP from MDA-MB-231 cells lysate, with anti-SHANK2 or anti-PRMT7 antibody, and the binding of PRMT7 and SHANK2 was examined by western blot. (**D**) Purified bacterially expressed GST or GST-PRMT7 was incubated with MDA-MB-231 cells lysate. GST-pulldown assay showed direct interaction between SHANK2 and recombinant PRMT7. (**E**) Diagram of the domains in SHANK2 protein. The schematics of the GST-SHANK2 expression plasmid, as well as domains and truncated mutants. (**F**) SHANK2 truncated mutants were incubated with MDA-MB-231 cells lysate. GST-pulldown assay showed direct interaction between PRMT7 and recombinant SHANK2. (**G**) HEK293T cells were transfected with increasing amounts of Flag-PRMT7 expression plasmids. Immunoprecipitation of SHANK2 with anti-SHANK2 antibody was performed. (**H**) MDA-MB-231 with or without stable expression of the indicated PRMT7 shRNA or a control shRNA. Immunoprecipitation of SHANK2 with anti-SHANK2 antibody was performed. (**I**) MDA-MB-231 cells with or without expressing PRMT7 shRNA and with or without reconstituted expression of WT PRMT7 or PRMT7 enzymatic activity mutant. Immunoprecipitation of SHANK2 with anti-SHANK2 antibody was performed. (**J**) HA-tagged SHANK2 was expressed in HEK293T cells. HA-purified SHANK2 protein was incubated with SAM and with or without purified bacterially expressed PRMT7. Methylation of recombinant SHANK2 protein was determined by western blot.

**Figure 1—figure supplement 1.** SHANK2 di-methylation was dependent on PRMT7. Immunoprecipitation and immunoblotting analyses were performed with the indicated antibodies. MDA-MB-231 cells expressing PRMT7 shRNA and with or without reconstituted expression of PRMT7 WT or PRMT7 R531K mutant. Immunoprecipitation of SHANK2 with anti-SHANK2 antibody was performed.

Next, we determine whether PRMT7 is involved in regulation of SHANK2 methylation. By using methylation assay, we found that overexpression of PRMT7 resulted in increased symmetric arginine di-methylation of SHANK2 in HEK293T cells (low level of PRMT7) (Figure 1G). In addition, we constructed lentiviral vectors containing shRNAs targeting the CDS of PRMT7 to knock down the endogenous PRMT7 of MDA-MB-231 cells. SHANK2 di-methylation level was reduced upon PRMT7 depletion, and the reduced di-methylation of SHANK2 was restored by the reconstituted expression of WT PRMT7 (PRMT7 WT) but not by mutant PRMT7 at its enzymatic domain (PRMT7 Mut) in MDA-MB-231 cells (high level of PRMT7) (Figure 1H and I). Meanwhile, SHANK2 di-methylation level was attenuated by the reconstituted expression of WT PRMT7 (PRMT7 WT) but not of mutant PRMT7 at its auto-methylation residue (PRMT7 R531 mutant) in PRMT7 depleted MDA-MB-231 cells (Figure 1—figure supplement 1). To further confirm PRMT7 directly methylated SHANK2, we used purified GST-PRMT7 and HA-SHANK2 for in vitro methylation assay followed by incubation with SAM (the methyl donor). Apparently, incubation of recombinant PRMT7 and SHANK2 gave rise to a remarkable increase in methylation of SHANK2 in the presence of SAM, while SHANK2 methylation was undetectable in the absence of SAM (Figure 1J). These results suggest that PRMT7 physically interacts with and methylates SHANK2.

### PRMT7 methylates SHANK2 at R240 residue

To further identify the methylation site of SHANK2, we performed mass spectrometric analysis using malignant breast cancer cell MDA-MB-231 lysate with overexpressed Rat HA-SHANK2 (a gift from Dr. Min Goo Lee). We identified that the arginine 240 residue (R240) of SHANK2 was di-methylated (Figure 2A). Using sequence homology comparison, we found that the R240 residue of SHANK2 is evolutionarily conserved (Figure 2B). To determine whether SHANK2 R240 residue was methylated by PRMT7, we constructed lentiviral vectors containing shRNAs targeting the 3’UTR of SHANK2 to knock down the endogenous SHANK2 of MDA-MB-231 cells. Then, we transfected SHANK2 wild-type or SHANK2 mutation with R240 residue replaced by lysine (SHANK2 R240K) into endogenous SHANK2 depleted MDA-MB-231 cells. We found that di-methylation level of SHANK2 R240K was lower when compared to SHANK2 WT in MDA-MB-231 cells (Figure 2C and D). We then overexpressed increasing doses of PRMT7 in HEK293T cells, and we found that SHANK2 R240 di-methylation level was increased accordingly (Figure 2E). PRMT5 has been reported to interact with PRMT7. We then examined the effect of PRMT5 overexpression on SHANK2 R240 di-methylation in HEK293T cells. We found that dosage dependent expression of PRMT5 did not increase the di-methylation at SHANK2 R240 (Figure 2—figure supplement 1A and B). Furthermore, we examined the effect of PRMT5 inhibitors (GSK591) on SHANK2 di-methylation (Fedoriw et al., 2019). We found that even when PRMT5 activity was inhibited, overexpression of PRMT7 could still increase the SHANK2 di-methylation level both in HEK293T and MDA-MB-231 cells (Figure 2—figure supplement 1C and D). Thus, although PRMT5 and PRMT7 existed in the same complex, our data indicated that di-methylation of SHANK2 R240 was mainly mediated by PRMT7. Taken together, these results indicate that PRMT7 physically interacts with SHANK2 to methylate R240 residue of SHANK2.

**Figure 2.** PRMT7 methylated SHANK2 at R240. (**A**) The purified SHANK2 from MDA-MB-231 cells transfected with HA-SHANK2 was analyzed for methylation by mass spectrometry. The SHANK2 R240 residue in fragmentation of KAARMRN was methylated. The Mascot score was 27.28, and the expectation value was 3.74E-04. (**B**) Alignment of the consensus SHANK2 sequences between different species near the R240 methylation site. (**C**) MDA-MB-231 cells with or without expressing SHANK2 shRNA and with or without reconstituted expression of WT SHANK2 or SHANK2 R240K mutant. Immunoprecipitation of HA with anti-HA antibody was performed. (**D**) Flag-tagged SHANK2 WT or SHANK2 R240K was transfected into MDA-MB-231 cells. HA-purified SHANK2 WT or SHANK2 R240K proteins were incubated with purified bacterially expressed PRMT7 and SAM. Methylation of SHANK2 protein was determined by western blot. (**E**) HEK293T cells were co-transfected with increasing amounts of Flag-PRMT7 and SHANK2 WT or SHANK2 R240K expression plasmids. Immunoprecipitation of SHANK2 with anti-SHANK2 antibody was performed.

**Figure 2—figure supplement 1.** The role of PRMT5 in PRMT7 mediated SHANK2 methylation. Immunoprecipitation and immunoblotting analyses were performed with the indicated antibodies. (**A**) HEK293T cells were co-transfected with control pcDNA3.1 or PRMT5 plasmids. Immunoprecipitation of SHANK2 with anti-SHANK2 antibody was performed. (**B**) HEK293T cells were co-transfected with increasing amounts of Flag-PRMT5 and SHANK2 WT or SHANK2 R240K expression plasmids. Immunoprecipitation of SHANK2 with anti-SHANK2 antibody was performed. (**C**) HEK293T cells with increasing amounts of Flag-PRMT7, PRMT5 and SHANK2 were treated with GSK591 (5 µM) or DMSO as control. Immunoprecipitation of HA with anti-HA antibody was performed. Western blot was performed with the indicated antibodies. (**D**) MDA-MB-231 cells with increasing amounts of Flag-PRMT7 were treated with GSK591 (5 µM) or DMSO as control. Immunoprecipitation of SHANK2 with anti-SHANK2 antibody was performed. Western blot was performed with the indicated antibodies.

### SHANK2 R240 methylation potentiates breast cancer cell migration and invasion

Previous reports showed that expression of *SHANK2* gene was higher in head and neck cancer tissues than that in adjacent tissues, and this upregulation was positively correlated with the survival rate and prognosis of the patients (Qin et al., 2016). Consistently, we also observed that *SHANK2* mRNA was highly expressed in human breast tumours (Figure 3A). To further investigate the clinical relevance of SHANK2 methylation with breast cancer, a direct western blot analysis of several subtypes of human breast cancer tumours was performed. The results demonstrated that SHANK2 methylation level was significantly higher in luminal B Her2^(+)^ and Triple-negative breast cancer samples, than that in normal, luminal A and luminal B Her2^(-)^ samples, which implicated a positive correlation between SHANK2 methylation and high metastatic potential (Figure 3B–E). In addition, to determine the relationship between PRMT7-mediated SHANK2 R240 methylation and metastasis, we analyzed the correlation between PRMT7 and the stage of breast cancer patients through TCGA Breast (BRCA) database. Among 1075 breast cancer patients, 89 out of 847 PRMT7 low-expression breast cancer patients were stage III or IV (10.5%), while 63 out of 228 PRMT7 high-expression breast cancer patients were stage III or IV (27.6%) (Figure 3—figure supplement 1). These data indicated that the expression of PRMT7 was positively correlated with the proportion of patients with stage III or IV breast cancer, which predicted poor prognosis. Next, we intended to study the effects of SHANK2 di-methylation on breast cancer cells. Out of 6 cell lines analyzed, high metastatic potential breast cancer cells (BT549 and MDA-MB-231) exhibited high SHANK2 di-methylation levels, whereas normal mammary epithelial cell (MCF10A), low metastatic potential breast cancer cell (MCF7, BT474 and T47D) showed relatively low SHANK2 di-methylation level (Figure 3F and G). Furthermore, we analyzed the expression profile of EMT-associated markers, and found that the epithelial marker ZO-1 was increased, while the mesenchymal markers Fibronectin and N-cadherin were decreased upon SHANK2 depletion; meanwhile, ZO-1 expression was decreased while Fibronectin and N-cadherin expressions were restored by reconstituted expression of SHANK2 WT but not of SHANK2 R240K in MDA-MB-231 and BT549 cells (Figure 3H and Figure 3—figure supplement 2A). However, SHANK2 did not induce EMT program in SHANK2 overexpressed MCF10A cells or in SHANK2 depleted MDA-MB-231 cells (Figure 3—figure supplement 2B and C). In addition, MMP2/MMP9 activation was inhibited by SHANK2 depletion, while the inhibition was abrogated by reconstituted expression of SHANK2 WT but not of SHANK2 R240K (Figure 3I), and the migration/invasion capabilities of MDA-MB-231 cells were also inhibited by SHANK2 depletion, and in both cases the inhibition was abrogated by reconstituted expression of SHANK2 WT but not of SHANK2 R240K (Figure 3J and K). Metastatic tumour cells are often accompanied by stem cell characteristics; however, we did not identify CD44^high^/CD24^low^ cell populations in SHANK2 depleting MDA-MB-231 or SHANK2-expressing MCF10A cells tested by FACS (Figure 3—figure supplement 2D). Together, these results strongly support the assumption that SHANK2 di-methylation is a crucial factor controlling EMT, migration and invasion characteristics of breast cancer cells.

**Figure 3.** SHANK2 R240 methylation promoted migration and invasion of breast cancer cells. (**A**) Comparison of SHANK2 expression level in breast cancer tissues of different breast cancer subtypes with that in normal tissues by RT-PCR. The logarithmic scale of 2^-ΔΔCt^ was used to measure the fold-change. β-actin was used as an internal reference. n = 27, *p<0.05, **p<0.01, ***p<0.001, one-way ANOVA test. (**B–E**) Comparison of PRMT7, SHANK2 and di-methylated SHANK2 levels in breast cancer tissues using western blot analysis. Data are based on the analysis of independent samples (n = 27). Immunoprecipitation of SHANK2 with anti-SHANK2 antibody was performed. *p<0.05, **p<0.01, ***p<0.001, ns = not significant, one-way ANOVA test. (**F**) SHANK2 mRNA expression in indicated breast cancer cell lines by RT-PCR. The logarithmic scale of 2^-ΔΔCt^ was used to measure the fold-change. β-actin was used as an internal reference. ***p<0.001, Student’s *t* test. (**G**) SHANK2 was IP from indicated breast cancer cell lines lysate, and input lysates and IP samples were analyzed using anti-methylation, anti-SHANK2 or anti-PRMT7 antibodies, as indicated. (**H**) MDA-MB-231 cells expressing SHANK2 shRNA and reconstituted expression of SHANK2 WT or SHANK2 R240K mutant. Western blot was performed with the indicated EMT marker antibodies. (**I**) MDA-MB-231 cells with or without stable expression of the indicated SHANK2 shRNA were transfected with SHANK2 WT or SHANK2 R240K mutant. Assessment of MMP2 and MMP9 enzymatic activities by gelatin zymography. (**J and K**) MDA-MB-231 cells expressing SHANK2 shRNA and reconstituted expression of SHANK2 WT or SHANK2 R240K mutant. Cell migration (**J**) and Invasion (**K**) were determined by transwell assays. (n = 3, independent experiments). Scale bars: 100 µm. Data represent the mean ± SD of three independent experiments. ***p<0.001, Student’s *t* test.

**Figure 3—figure supplement 1.** PRMT7 was associated with clinical outcomes. Correlation between PRMT7 expression and clinical outcomes through analysis of stage of breast cancer patients in TCGA Breast (BRCA) database(n = 1075 patients). **p<0.01, Chi2 test.

**Figure 3—figure supplement 2.** SHANK2 was involved in breast cancer cells EMT. (**A**) BT549 cells with or without expressing SHANK2 shRNA and with or without reconstituted expression of SHANK2 WT or SHANK2 R240K mutant. Western blot was performed with the indicated EMT marker antibodies. (**B**) MDA-MB-231 with or without stable expression of the indicated SHANK2 shRNA or a control shRNA. Western blot was performed with the indicated EMT marker antibodies. (**C**) MCF10A cells expressing the indicated HA-tagged SHANK2. Western blot was performed with the indicated EMT marker antibodies. (**D**) Stem-like CD44^high^/CD24^low^ profile in MDA-MB-231 cells transfected with stable expression of the indicated SHANK2 shRNA or a control shRNA, and MCF10A cells expressing the indicated HA-tagged SHANK2.

### R240 methylation disturbs SPN-ANK domain blockade of SHANK2

To explore the mechanism of SHANK2 methylation in breast cancer cell migration and invasion, we studied the conformational changes of wild-type SHANK2 (WT), di-methylated SHANK2 at R240 (Dimethyl R240), and its mutant (R240K) by using molecular dynamics simulations (Kumar et al., 1992; Phillips et al., 2005; Vanommeslaeghe et al., 2010; Zhu and Hummer, 2012; Huang and MacKerell, 2013; Wang et al., 2016; Waterhouse et al., 2018; Grossfield, 2020). As shown in Figure 4A, the SPN domain in Dimethyl R240 needs less energy to reach an ‘open’ state than that in SHANK2 WT and R240K, according to the free energy profile. To further investigate how the dimethylated R240 affects the conformational changes between SPN and ANK domains, the trajectory for the window with the global minimum free energy (the distance between SPN and ANK is 31.5 Å, the SPN and ANK domains were represented in different colours in Figure 4B) in WT, the one (the distance between SPN and ANK is 32 Å) in Dimethyl R240 and the one (the distance between SPN and ANK is 30 Å) in R240K were analysed. R240 can form hydrogen bonds with its neighbouring residue H236 and by this R240 remotely influences the interactions between SPN and ANK via hydrogen bond network (Figure 4C and D). It indicates that R240 methylation dramatically decreased interactions between R240 and H236. It further weakened the stability of the closed state of SHANK2. Thus, structural analyses suggest that SHANK2 R240 methylation disrupted SPN-ANK domain blockade to ‘open’ SHANK2, providing more chances for insertion of partner proteins.

**Figure 4.** R240 methylation impaired SPN-ANK domain interaction of SHANK2. (**A**) Definition of the SPN domain (coloured in green) and the ANK domain (coloured in cyan) in SHANK2. The location of R240 was represented with sticks. (**B**) Key residues forming hydrogen bonds between SPN and ANK in SHANK2 WT. R240 can form hydrogen bonds with H236 in ANK (coloured in magenta). (**C**) Key residues forming hydrogen bonds between SPN and ANK in SHANK2 R240K. K240 can still form hydrogen bonds with H236 in ANK (coloured in magenta). (**D**) Potential of mean forces for the conformational changes (from closed state to the open state) of SPN and ANK in the wild type (WT, black line), methylated (Dimethyl R240, blue line) and mutant (R240K, red line) SHANK2.

### SHANK2 R240 methylation recruits FAK/dynamin2/talin complex to endosome

A previous study reported that SHANK3 SPN domain interacts with the ANK domain in an intramolecular manner, thereby restricting access of either Sharpin or α-fodrin (Mameza et al., 2013). To further figure out which SHANK2-bound proteins might be affected by SHANK2 R240 methylation induced structural changes, we used mass spectrometry to find the possible regulatory factors. The mass spectrometric data showed that SHANK2 could interact with numerous endosome associate proteins, including β1-integrin, talin, FAK, EEA1, dynamin2, clathrin, AP2 and cortactin (Figure 5A,B and Figure 5—figure supplement 1A), suggesting that methylated SHANK2 might contribute to endosome formation. To test this hypothesis, we first verified the mass spec data by using CoIP assays and we confirmed that talin, FAK, dynamin2, cortactin and SHANK2 were in the same complex in MDA-MB-231 cells (Figure 5C). To determine whether PRMT7-mediated SHANK2 methylation is involved in regulation of endocytosis, we overexpressed PRMT7 in MCF7 cells (low level of PRMT7). We found that overexpression of PRMT7 promoted the co-precipitation of dynamin2/talin/FAK/SHANK2 with cortactin in MCF7 cells, and the interaction was reduced in PRMT7 depleted MDA-MB-231 cells (Figure 5D and F). Meanwhile, the PRMT7 enzymatic activity mutation (PRMT7 Mut) and PRMT7 R531 mutant attenuated the formation of dynamin2/talin/FAK/SHANK2/cortactin complex in PRMT7 depleted MDA-MB-231 cells (Figure 5—figure supplement 1B and C). Additionally, overexpression of PRMT7 triggered an accumulation in the number of EEA1-positive endosomes with more talin, FAK, EEA1 and dynamin2 colocalization in MCF7 cells, and the colocalization was attenuated in PRMT7 depleted MDA-MB-231 cells (Figure 5E and G). Consistently, the formation of dynamin2/talin/FAK/SHANK2/cortactin was significantly increased by reconstituted expression of SHANK2 WT but not of SHANK2 R240K in SHANK2 depleted MDA-MB-231 cells (Figure 5H). Meanwhile, SHANK2 WT promoted the recruitment of EEA1-positive endosomes and the majority of SHANK2 was associated with endosome associate proteins, which was significantly reduced by SHANK2 R240K in MDA-MB-231 and BT549 cells (Figure 5I and Figure 5—figure supplement 1D). Consistent with this finding, the interaction of dynamin2/talin/FAK/SHANK2/cortactin and the localization between talin, FAK, EEA1 and dynamin2 with endosome compartment was enhanced by reconstituted expression of SHANK2 R240F (as a methyl-mimic) but not of SHANK2 WT or SHANK2 R240K in MCF10A cells expressing low level of PRMT7 (Figure 5J and K). To assess the requirement of SHANK2 in PRMT7-induced interaction between talin and FAK, we silenced SHANK2 by shRNA in PRMT7-MCF7 cells. SHANK2 silencing partially reduced the formation of dynamin2/talin/FAK/SHANK2/cortactin complex (Figure 5—figure supplement 2A) and markedly decreased the interaction between talin and FAK (Figure 5—figure supplement 2B). Together, our data suggest that SHANK2 R240 di-methylation catalysed by PRMT7 is in favour of the assembly of a multi-protein complex to facilitate endosome formation.

**Figure 5.** SHANK2 R240 methylation promotes FAK/dynamin2/talin complex co-localized with endosome. (**A**) SHANK2 associated proteins from HA-SHANK2 expressing stable MDA-MB-231 cells were immunopurified with anti-HA (α-HA) affinity resins. The protein bands were analyzed by mass spectrometry. (**B**) Representative peptide fragments of SHANK2 associated proteins and peptide coverage of the indicated proteins are shown. (**C**) Endogenous talin, FAK, dynamin2, EEA1 and SHANK2 were IP from MDA-MB-231 cells, with indicated antibodies, and the binding of talin, FAK, dynamin2 and SHANK2 was examined by western blot. (**D**) MCF7 cells with expression of the indicated Flag-Vector or Flag-tagged PRMT7. Immunoprecipitation of cortactin with anti-cortactin antibody was performed. (**E**) Confocal images of PRMT7, dynamin2, SHANK2, EEA1, talin, Rab5, FAK, cortactin and DAPI staining in MCF7 cells with expression of the indicated Flag-Vector or Flag-tagged PRMT7. Scale bars, 10 µm. (**F**) MDA-MB-231cells with or without stable expression of the indicated PRMT7 shRNA or a control shRNA. Immunoprecipitation of cortactin with anti-cortactin antibody was performed. (**G**) confocal images of PRMT7, dynamin2, SHANK2, EEA1, talin, Rab5, FAK, cortactin and DAPI staining in MDA-MB-231cells with or without stable expression of the indicated PRMT7 shRNA or a control shRNA. Scale bars, 10 µm. (**H**) MDA-MB-231cells expressing SHANK2 shRNA with or without reconstituted expression of WT SHANK2 or SHANK2 R240K mutant. Immunoprecipitation of cortactin with anti-cortactin antibody was performed. (**I**) Confocal images of PRMT7, dynamin2, SHANK2, EEA1, talin, Rab5, FAK, cortactin and DAPI staining in MDA-MB-231cells expressing SHANK2 shRNA with or without reconstituted expression of WT SHANK2 or SHANK2 R240K mutant. Scale bars, 10 µm. (**J**) MCF10A cells with reconstituted expression of SHANK2 WT, SHANK2 R240K or SHANK2 R240F (arginine to phenylalanine) mutant. Immunoprecipitation of SHANK2 with anti-SHANK2 antibody was performed. (**K**) Confocal images of PRMT7, dynamin2, SHANK2, EEA1, talin, Rab5, FAK, cortactin in MCF10A cells with reconstituted expression of SHANK2 WT, SHANK2 R240K or SHANK2 R240F mutant. Scale bars, 10 µm.

**Figure 5—figure supplement 1.** SHANK2 was essential for the interaction and activity between talin and FAK. Immunoprecipitation and immunoblotting analyses were performed with the indicated antibodies. (**A**) Representative peptide fragments of SHANK2 associated proteins and peptide coverage of the indicated proteins are shown. (**B**) MDA-MB-231 cells expressing PRMT7 shRNA and with or without reconstituted expression of WT PRMT7 or PRMT7 enzymatic activity mutant. Immunoprecipitation of SHANK2 with anti-SHANK2 antibody was performed. (**C**) MDA-MB-231 cells expressing PRMT7 shRNA and with or without reconstituted expression of PRMT7 WT or PRMT7 R531K mutant. Immunoprecipitation of cortactin with anti-SHANK2 antibody was performed. (**D**) BT549 cells with or without expressing SHANK2 shRNA and with or without reconstituted expression of SHANK2 WT or SHANK2 R240K mutant. Immunoprecipitation of cortactin with anti-SHANK2 antibody was performed.

**Figure 5—figure supplement 2.** SHANK2 was necessary for the interaction between talin and FAK. (**A**) MCF7 cells with reconstituted expression of PRMT7 and with or without stable expression of the indicated SHANK2 shRNA. Immunoprecipitation of cortactin with anti-cortactin antibody was performed. (**B**) MCF7 cells with reconstituted expression of PRMT7 and with or without stable expression of the indicated SHANK2 shRNA. Immunoprecipitation of FAK with anti-FAK antibody was performed.

**Figure 5—figure supplement 3.** SHANK2 was co-localized with exosome markers. (**A**) confocal images of SHANK2, CD63, CD81 and DAPI staining in MDA-MB-231cells expressing SHANK2 shRNA with or without reconstituted expression of WT SHANK2 or SHANK2 R240K mutant. Scale bars, 10 µm. (**B**) confocal images of EEA1, CD63, CD81 and DAPI staining in MDA-MB-231cells expressing SHANK2 shRNA with or without reconstituted expression of WT SHANK2 or SHANK2 R240K mutant. Scale bars, 10 µm. .

### SHANK2 R240 methylation activates endosomal FAK signalling

Persistent activation of FAK signalling on endosomes promotes cancer cell dissemination (Alanko and Ivaska, 2016). To determine whether SHANK2 methylation was involved in endosomal FAK pathway activation, we examined phosphorylation of FAK and its downstream cortactin signalling cascade. As expected, overexpression of PRMT7 markedly increased FAK and cortactin phosphorylation in MCF7 cells, and PRMT7 depletion profoundly decreased FAK and cortactin phosphorylation in MDA-MB-231 cells (Figure 6A and B). Consistently, FAK and cortactin were activated by reconstituted expression of SHANK2 WT but not of SHANK2 R240K (Figure 6C). Furthermore, blocking FAK activation with FAK inhibitor GSK2256098 did inhibit phosphorylation of FAK and cortactin upregulated by SHANK2 R240F in SHANK2 depleted MDA-MB-231 cells (Figure 6D). The similar results were also observed in MCF10A cells co-transfected with SHANK2 R240F and FAK WT, but not with SHANK2 WT or SHANK2 R240K and FAK Y397K (Figure 6E and Figure 6—figure supplement 1A–C). Consistently, we found that SHANK2 R240F or SHANK2 WT, but not SHANK2 R240K increased phosphorylation of FAK and cortactin in SHANK2 depleted MDA-MB-231 cells (Figure 6F). To determine if PRMT7-dependent SHANK2 methylation responsible for FAK activation was dependent on endocytosis, MDA-MB-231-SHANK2 depletion cells with reconstituted expression of SHANK2 R240F were treated with the dynamin inhibitor-dynasore. Treatment with dynasore or silencing of EEA1 greatly decreased SHANK2 R240F induced-phosphorylation of FAK and cortactin in MDA-MB-231 cells (Figure 6F and G). FAK activation was also thought to inhibit apoptosis for cancer cell dissemination. We found that apoptotic cells were increased upon reconstituted expression of SHANK2 R240K but not of SHANK2 WT (Figure 6—figure supplement 1D). Collectively, these findings provide evidence that SHANK2 di-methylation mediated by PRMT7 potentiates FAK and cortactin activation through activating endocytosis.

**Figure 6.** SHANK2 R240 methylation activated endosomal FAK signals. (**A**) Phosphorylated/total FAK and cortactin were determined in MCF-7 cells expressing the indicated Flag-tagged PRMT7. Western blot was performed with the indicated antibodies. (**B**) Phosphorylated/total FAK and cortactin were determined in MDA-MB-231 cells with or without stable expression of the indicated SHANK2 shRNA or a control shRNA. Western blot was performed with the indicated antibodies. (**C**) Phosphorylated/total FAK and cortactin were determined in MDA-MB-231 cells with or without expressing SHANK2 shRNA and with or without reconstituted expression of WT SHANK2 or SHANK2 R240K mutant. Western blot was performed with the indicated antibodies. (**D**) Phosphorylated/total FAK and cortactin were determined in MDA-MB-231 cells expressing SHANK2 shRNA with or without reconstituted expression of WT SHANK2 or SHANK2 R240K or SHANK2 R240F mutant, SHANK2 R240F were treated with GSK2256098 (10 µM) or DMSO as control. Western blot was performed with the indicated antibodies. (**E**) Phosphorylated/total FAK and cortactin were determined in MCF10A cells co-transfected with SHANK2 and/or FAK plasmids. Western blot was performed with the indicated antibodies. (**F**) Phosphorylated/total FAK and cortactin were determined in MDA-MB-231 cells expressing SHANK2 shRNA with or without reconstituted expression of WT SHANK2, SHANK2 R240K or SHANK2 R240F mutant. SHANK2 R240F group was treated with dynasore (80 µM) or DMSO as control. Western blot was performed with the indicated antibodies. (**G**) Phosphorylated/total FAK and cortactin were determined in MDA-MB-231 cells expressing SHANK2 shRNA with or without reconstituted expression of WT SHANK2, SHANK2 R240K or SHANK2 R240F mutant. SHANK2 R240F with or without stable expression of the indicated EEA1 shRNA or a control shRNA. Western blot was performed with the indicated antibodies.

**Figure 6—figure supplement 1.** SHANK2 R240F activated FAK and cortactin. (**A**) Phosphorylated/total FAK and cortactin were determined in MCF10A cells co-transfected with SHANK2 and/or cortactin plasmids. Western blot was performed with the indicated antibodies. (**B**) MCF10A cells co-transfected with SHANK2 and/or cortactin plasmids. Assessment of MMP9 enzymatic activities by gelatin zymography. (**C**) MCF10A cells co-transfected with SHANK2 and/or cortactin plasmids. Assessment of the MMP9 enzymatic activities by gelatin zymography. (**D**) MDA-MB-231 cells with or without expressing SHANK2 shRNA and with or without reconstituted expression of SHANK2 WT or SHANK2 R240K mutant. Flow cytometric analysis of annexin V-FITC/PI staining was conducted to examine cell death.

### SHANK2 R240 methylation promotes migration and invasion through activating endosomal signals

Thus far, we have found that the PRMT7-mediated SHANK2 R240 methylation triggered breast cancer cell migration/invasion, and SHANK2 R240 methylation promoted endocytosis and endosomal FAK activation. We next wonder if the SHANK2 methylation-promoted migration and invasion is dependent on the activation of endosomal signals. Indeed, treatment with dynasore decreased PRMT7 induced-EMT program and migration/invasion capabilities of MCF7 cells (Figure 7A–C). Likewise, EMT and cell migration/invasion were activated by reconstituted expression of SHANK2 R240F or SHANK2 WT but not of SHANK2 R240K in SHANK2-depleted MDA-MB-231 cells (Figure 7D–F). To determine the functional role of SHANK2 R240 methylation is dependent on endocytosis, we treated SHANK2 R240F MDA-MB-231 cells with dynasore, and found that dynasore dramatically inhibited the effects of SHANK2 R240F induced-EMT and cell migration/invasion (Figure 7D–F). Since multiple endosomal signalling pathways are EEA1 dependent, we silenced EEA1 to test the impact of SHANK2 R240 methylation on EMT program and migration/invasion capabilities. Similarly, knockdown of EEA1 also markedly reduced SHANK2 R240F induced-EMT and cell migration/invasion (Figure 7G–I). Since SHANK2 R240 methylation promotes cell migration/invasion through activating endosomal FAK signalling, we treated SHANK2 R240F MDA-MB-231 cells with FAK inhibitor GSK2256098, and found that GSK2256098 also inhibited the effects of SHANK2 R240F induced-EMT and cell migration/invasion (Figure 7J–L). Taken together, these results indicate that the PRMT7-induced SHANK2 R240 methylation triggers breast cancer cell migration and invasion through activating endosomal FAK signalling.

**Figure 7.** SHANK2 R240 methylation promoted migration and invasion of breast cancer cells by activating endosomal FAK signals. (**A**) MCF7cells expressing the indicated Flag-tagged PRMT7. MCF7-Vector and MCF7-PRMT7 groups were treated with dynasore (80 µM) or DMSO as control. Western blot was performed with the indicated EMT marker antibodies. (**B and C**) MCF7 cells expressing the indicated Flag-tagged PRMT7. MCF7-Vector and MCF7-PRMT7 groups were treated with dynasore (80 µM) or DMSO as control. Cell migration (**B**) and Invasion (**C**) were determined by transwell assays. (n = 3, independent experiments). Scale bars: 50 µm. Data represent the mean ± SD of three independent experiments. Scale bars,100 µm. ***p<0.001, Student’s *t* test. (**D**) MDA-MB-231 cells expressing SHANK2 shRNA with or without reconstituted expression of WT SHANK2, SHANK2 R240K or SHANK2 R240F mutant. SHANK2 R240F group was treated with dynasore (80 µM) or DMSO as control. Western blot was performed with the indicated EMT marker antibodies. (**E and F**) MDA-MB-231 cells expressing SHANK2 shRNA with or without reconstituted expression of WT SHANK2, SHANK2 R240K or SHANK2 R240F mutant. SHANK2 R240F group was treated with dynasore (80 µM) or DMSO as control. Cell migration (**E**) and Invasion (**F**) were determined by transwell assays. (n = 3, independent experiments). Scale bars: 100 µm. ***p<0.001, Student’s *t* test. (**G**) MDA-MB-231 cells expressing SHANK2 shRNA with or without reconstituted expression of WT SHANK2, SHANK2 R240K or SHANK2 R240F mutant. SHANK2 R240F with or without stable expression of the indicated EEA1 shRNA or a control shRNA. Western blot was performed with the indicated EMT marker antibodies. (**H and I**) MDA-MB-231 cells expressing SHANK2 shRNA with or without reconstituted expression of WT SHANK2, SHANK2 R240K or SHANK2 R240F mutant. SHANK2 R240F with or without stable expression of the indicated EEA1 shRNA or a control shRNA. Cell migration (**H**) and Invasion (**I**) were determined by transwell assays. (n = 3, independent experiments). Scale bars: 100 µm. ***p<0.001, Student’s *t* test. (**J**) MDA-MB-231 cells expressing SHANK2 shRNA with or without reconstituted expression of WT SHANK2, SHANK2 R240K or SHANK2 R240F mutant. SHANK2 R240F group was treated with GSK2256098 (10 µM) or DMSO as control. Western blot was performed with the indicated EMT marker antibodies.

### SHANK2 R240 methylation promotes breast cancer metastasis through elevating endosomal FAK activation

The above findings intrigued us to test the functions of SHANK2 R240 methylation in the pathological progression of breast cancer. To assess the biological effects of SHANK2 R240 methylation in vivo, we examined whether SHANK2 di-methylation affected tumour metastasis in xenograft mouse models. We injected equal amounts of MDA-MB-231-scramble cells, MDA-MB-231-SHANK2 depletion cells, MDA-MB-231-SHANK2 depletion cells with reconstituted expression of SHANK2 WT, SHANK2 R240K or SHANK2 R240F into the vail veins of female nude BALB/c nude mice, and mice bearing SHANK2 R240F were treated with or without FAK inhibitor GSK2256098. The results demonstrated that lung metastases and the number of metastatic pulmonary nodules were dramatically decreased by reconstituted expression of SHANK2 R240K, but not of SHANK2 WT or SHANK2 R240F (Figure 8A). We also discovered that the mice injected with SHANK2 R240F cells and treated with GSK2256098 formed fewer lung metastatic foci than that injected with SHANK2 R240F (Figure 8B). In addition, immunohistochemistry staining results indicated that SHANK2 R240F expression reinforced FAK Y397 and cortactin Y421 phosphorylation, whereas SHANK2 R240F with GSK2256098 treatment profoundly inhibited SHANK2 R240F induced-FAK Y397 and cortactin Y421 phosphorylation (Figure 8C and D). Our observations indicate that SHANK2 di-methylation induces metastasis of MDA-MB-231 cells in vivo through activating FAK signalling. Likewise, we analyzed 27 human primary breast cancer specimens (Figure 3A and B) with PRMT7, p-FAK and p-cortactin antibody. Immunohistochemistry staining results revealed a correlation among PRMT7, FAK Y397 and cortactin Y421 phosphorylation levels, and the clinical aggressiveness of breast cancer (Figure 8E,F and Figure 8—figure supplement 1). Together, these data indicate that SHANK2 R240 methylation promotes breast cancer metastasis through activating FAK signalling.

**Figure 8.** Arginine methylation at SHANK2 R240 promoted metastasis through activates FAK signalling. (**A**) Equal numbers of MDA-MB-231 cells expressing SHANK2 shRNA with or without reconstituted expression of WT SHANK2, SHANK2 R240K or SHANK2 R240F mutant. SHANK2 R240F group was treated with GSK2256098 or DMSO. Cells were tail-vein injected into BALB/c nude mice, and lung metastasis was determined. The gross appearance of the lungs and the tumour nodules on the lungs were examined. Tumours were paraffin embedded and stained with H and E at Day12. n = 5 tumours in each group. IHC analyses of tumour tissues were performed with anti-p-FAK or anti-p-cortactin antibody. Scale bars,100 µm. (**B**) The number of visible surface metastatic lesions in lungs was counted. (n = 5 mice for each group, **p<0.01, ***p<0.001, ns = not significant, one-way ANOVA test). (**C, D**) p-FAK and p-cortactin -positive cells were quantified in 10 microscope fields. **p<0.01, ***p<0.001, ns = not significant, one-way ANOVA test. (**E, F**) Typical pictures of the immunohistochemical staining of PRMT7, p-FAK and p-cortactin in breast cancer samples. Scale bars,100 µm. n = 27, **p<0.01, Student’s t test.

**Figure 8—figure supplement 1.** PRMT7 was associated with III stage breast cancer. (**A**) Typical pictures of the immunohistochemical staining of PRMT7, p-FAK and p-cortactin in breast cancer samples. Scale bars,100 µm. (**B–E**) Statistic of stage and staining correlates with subtype. n = 27, ***p<0.001, Chi2 test.

## Discussion

Protein arginine methylation modification is involved in a variety of cellular biological events, such as epigenetic gene activation/repression, alternative mRNA splicing, DNA repair and immune surveillance (Jarrold and Davies, 2019). Recent reports showed that endocytosis activity required methionine and PRMT1 (Albrecht et al., 2018). Nevertheless, the roles and mechanisms of arginine methylation in regulation of cell endocytosis remain poorly defined. In this study, we report a new substrate of PRMT7, the scaffold protein SHANK2, which is di-methylated at arginine 240 residue to maintain endocytic activity. In particular, SHANK2 R240K methylation disturbs SPN-ANK domain blockade of SHANK2, thereby resulting in the accumulation of dynamin2, talin, FAK and cortactin on the endosome. SHANK2 R240 methylation further activates endosomal FAK/cortactin signals, which increases the migration of SHANK2-dependent breast cancer metastasis. (Figure 9).

**Figure 9.** A model for PRMT7-mediated SHANK2 methylation that promotes breast cancer migration through activating endosomal FAK signalling In the absence of PRMT7, SHANK2 cannot interact with dynamin2/talin/FAK/cortactin complex to endosome. In the presence of PRMT7, R240-methylated SHANK2 disturbs SPN-ANK domain blockade of SHANK2, thereby promoting the co-localization of dynamin2/talin/FAK/cortactin complex on endosome, further activating FAK signalling to promote tumour cells migration.

Cancer cells are highly compartmentalized by the endomembrane system, which is functionally defined by the scaffold proteins dynamin, EEA1 or APPL1 (Sandra, 2017). Our mass spectrometry results suggested that methylated SHANK2 not only interacted with talin, FAK and cortactin, but also with endosome associate proteins such as clatharin, AP-2 and dynamin2 (Figure 5B). It is implicated that the methylated SHANK2 might be involved in clatharin-mediated endocytosis. Dynamin is best known for its role in catalyzing membrane scission at late stages of clathrin-mediated endocytosis to release clathrin-coated vesicles into the cytosol (Kaksonen and Roux, 2018). Furthermore, increasing evidence suggests that dynamin can also regulate earlier stages of endosome maturation through binding the scaffold protein EEA1, in turn regulate the recruitment of other factors to the membrane that control endosomal sorting and maturation (Hamidi and Ivaska, 2018). Our results demonstrated that PRMT7 promoted dynamin2 interaction with methylated SHANK2 (Figure 5H). Moreover, the PRMT7-mediated SHANK2 methylation rendered EEA1 to co-localize with SHANK2 (Figure 5I). These results indicate that methylated SHANK2 might enhance the activity of dynamin2 and thus regulate the formation of endosome.

Scaffold proteins SHANK1, 2, three are able to bind and interact with a wide range of proteins including actin binding proteins and actin modulators, such as dynamin2, cortactin, RICH2, and PIX (Lee et al., 2010; Sheng and Kim, 2000). SHANK1, 2, three have been reported to affect the structure and function of the neural circuits and to regulate autism spectrum disorders; but their roles in tumourigenesis are far from illuminated. Recent studies reported that SHANK1 and SHANK3 acted as negative regulators of integrin activity by binding R-Ras, thereby inhibiting migration and invasion of MDA-MB-231 cells (Lilja et al., 2017). In contrast to SHANK1 and SHANK3, the present study revealed that SHANK2, especially the methylated SHANK2, was correlated with high level of incidence of breast cancer (Figure 3B). Our data demonstrated that methylated SHANK2 promoted breast cancer metastasis (Figure 8A). Like SHANK3, our mass spectrometry results demonstrated that methylated SHANK2 could bind to receptor proteins, not only integrin but also Met, NRP1 and EGFR, which indicated that PRMT7-SHANK2 might be involved in receptor mediated endocytosis (Figure 5—figure supplement 1A). Although several studies reported that SHANK2 and SHANK3 could form heterodimers, our mass spectrometry results did not found SHANK1 or SHANK3 interacting with SHANK2. Moreover, by comparing SHANK3 protein sequence with SHANK2, we did not find the conservative RXR motif that was a potential methylation sequence by PRMT7. Therefore, whether SHANK3 and SHANK2 have crosstalk still needs further study.

The intracellular trafficking of endosome must be tightly controlled in space and time to enable effective cell adhesion and microenvironmental sensing and compartmentalize it from other cellular processes. Organelles of these intracellular trafficking pathways—including endosomes, lysosomes, exosome, the endoplasmic reticulum (ER), the Golgi apparatus, and the plasma membrane are coupled by clatharin-dependent membrane vesicles delivery. In our study, we also demonstrated that methylated SHANK2 could interact with relative endomembrane organelles marker, such as EEA1, LAMP1, Calnexin, GOLM1, Ninein, CD63, TOM70 and LanminA/C (Figure 5—figure supplement 1A). These results indicated that SHANK2 could localize not only on endosomes but also on lysosome, mitochondria, ER, Golgi, centrosome, exosome and nuclear. Exosomes are key mediators of intercellular communication and can be detected in the tumour microenvironment. Although a small amount of the cell surface SHANK2 was detected, it was barely detected on plasma membrane by immunofluorescence analysis (Figure 5L). These data suggested that SHANK2 was rapidly internalized after recycling back to the cell surface and/or they might transport to the extracellular space by secreted exosomes. Exosomes are vesicles derived from late endosomes, also known as multivesicular bodies, and can be secreted to the extracellular environments by most cell types. Indeed, we found that the methylated SHANK2 was co-localized with several common exosome marker proteins, including CD63 and CD81 (Figure 5—figure supplement 3A). Meanwhile, SHANK2 WT promoted recruitment of EEA1-positive endosomes and co-localized more CD63 and CD81 than that of SHANK2 R240K in MDA-MB-231 cells (Figure 5—figure supplement 3B). Thus, it is likely that the PRMT7-SHANK2 might be secreted by exosomes and continuously internalized and sustained the active talin/FAK/cortactin complexes on endosomes, and thereby provided persistent endosomal signals for tumour progression.

In conclusion, data presented in this report outlines a working model in which PRMT7 regulates breast tumour metastasis by methylating SHANK2, a new substrate of PRMT7. Specifically, SHANK2 methylation enforces tumour metastasis, while it simultaneously promotes breast cancer cell migration and invasion via triggering endosomal FAK signal activation (Figure 9). As a key player in breast cancer development, methylated SHANK2 might be a potential therapeutic target.

## Materials and methods

### Cell lines and reagents

MCF10A, MCF7, T47D, BT474, MDA-MB-231, BT549 and HEK293T cell lines were purchased from ATCC, where all the cell lines were characterized by DNA finger printing and isozyme detection. Cells were immediately expanded and frozen such that they could be revived every 3 to 4 months. Cells were tested every 6 months to ensure negative for mycoplasma contamination with Lonza MycoAlert Mycoplasma Detection Kit (LT07-218, Lonza, Basel, Switzerland). All cell lines were mycoplasma negative. Cell lines were authenticated using Short Tandem Repeat (STR) analysis as described in 2012 in ANSI Standard (ASN-0002) by the ATCC Standards Development Organization (SDO). MCF10A cells were were cultured in DMEM/F12 supplemented with 20 ng/ml EGF (Sigma-Aldrich, E9644), 0.5 mg/ml hydrocortisone (Sangon, A610506), 100 ng/ml cholera toxin (Sigma-Aldrich, C8180), 10 mg/ml insulin (Gibco, Grand Island, NY, USA, 12585–014), hFGF basic (R and D Systems, Minneapolis, MN, USA, P09038), 10 U/ml penicillin-streptomycin, and 5% horse serum (Gibco), and incubated at 37°C in 5% CO2. BT549, BT474 and T47D cells were cultured in RPMI-1640 medium supplemented with 10% FBS (ExCell Bio). MDA-MB-231 cells were cultured in L15 medium with 10% FBS at 37°C without CO_2_; HEK293T and MCF7 cells were cultured in DMEM containing 10% FBS. Dynasore (S8047), GSK591 (S8111), GSK2256098 (S5823) were purchased from Selleck Chemicals.

### Antibodies and plasmids

The following antibodies were used: antibodies against N-cadherin (561553, 1:1000 for WB, BD Biosciences), fibronectin (610077, 1:1000 for WB, BD Biosciences), β-catenin (610154, 1:1000 for WB, BD Biosciences), EEA1 (610456, 1:100 for IF, BD Biosciences), Rab5 (610724, 1:100 for IF, BD Biosciences), β-actin (A5228, A1978, 1:5000 for WB, Sigma-Aldrich), HA (H9658, 1:1000 for WB and 1:200 for IP, Sigma-Aldrich), MMP2 (GTX-104577, 1:1000 for WB, GeneTex), MMP9 (40086, 1:1000 for WB, GeneTex), p-cortactin (BS4778, 1:100 for IHC, bioworld), p-cortactin (ab47768, 1:1000 for WB, Abcam), mono methyl Arginine (ab415, 1:500 for WB, Abcam), asymmetric dimethyl Arginine (ab412, 1:500 for WB, Abcam), Dyn2 (ab3457, 1:100 for IF and 1:1000 for WB, Abcam), Flag (m20008, 1:1000 for WB and 1:200 for IP, Abmart), p-FAK (700255, 1:200 for IHC, Invitrogen), PRMT7 (sc-376077, 1:200 for IHC, santa cruz), PRMT7 (14762S, 1:200 for IP, 1:100 for IF and 1:1000 for WB, cell signaling technology), SHANK2 (#12218, 1:100 for IF, 1:200 for IP and 1:500 for WB, cell signaling technology), p-FAK (#8556, 1:1000 for WB, cell signaling technology), FAK (#3285, 1:1000 for WB and 1:100 for IF, cell signaling technology), p-talin (#13589, 1:1000 for WB, cell signaling technology), talin (#4021, 1:1000 for WB and 1:100 for IF, cell signaling technology), ZO-1 (#5406S, 1:1000 for WB, cell signaling technology), symmetric dimethyl Arginine (SYM10, 1:500 for WB, Millipore), PRMT5 (2882018, 1:1000 for WB, Millipore), cortactin (05–180, 16–228, 1:1000 for WB and 1:100 for IF, Millipore).

Flag-cortactin expression vector was a gift from Dr. Alpha S. Yap (Division of Cell Biology and Molecular Medicine, The University of Queensland, Australia), HA-SHANK2 expression vector was a gift from Dr. Min Goo Lee (Department of Pharmacology, Pusan National University, Pusan, Korea), pcDNA3-HA-SHANK2, pWPXLD-SHANK2, pWPXLD-Flag-PRMT7, pWPXLD-Flag-PRMT5, pWPXLD-PRMT5. Additionally, shSHANK2#1 and shSHANK2#2 oligonucleotides were designed and cloned into lentiviral RNAi system pLKO.1. The sequences of shRNAs, which were designed to target human genes, were described below.

shPRMT7#1: GGAACAAGCTATTTCCCATCC (targeting CDS region).
shPRMT7#2: GGATGCAGTGTGTGTACTTCC (targeting CDS region).
shSHANK2#1: GGAGTTAGTCAAAGCACAAAG (targeting CDS region).
shSHANK2#2: GCTTGGAGCAAGAGAGAATTT (targeting 3’UTR region).
shEEA1#1: GCGGAGTTTAAGCAGCTACAA (targeting CDS region).

### Western blotting and immunoprecipitation

Immunoprecipitation was performed with the lysates from indicated cultured cells and followed by the immunoblotting with corresponding antibodies. Briefly, the cells were collected and washed three times with cold PBS. Cells were harvested and lysed in buffer A [20 mM Tris-HCl (pH 8.0), 10 mM NaCl, 1 mM EDTA, and 0.5% NP-40] plus a protease inhibitor and phosphatase inhibitor cocktails (Roche Diagnostics, Indianapolis, IN, USA) for 30 min at 4°C. The supernatant was subjected to SDSPAGE, transferred to PVDF (EMD-Millipore) and detected by ECL reagents (GE Healthcare, Buckinghamshire, United Kingdom).

### RNA extraction, reverse transcription and real-time RT-PCR

Total RNA was extracted using Trizol reagent (TaKaRa, Dalian, China), according to the manufacturer’s instructions. RT-PCR was performed using the Access RT-PCR System from Promega. Real-time PCR was done using SYBR Green Realtime PCR Master Mix (TOYOBO, Osaka, Japan) on a LightCycler 480 Real Time PCR system (Roche).

### The β-actin was used as an internal control. The sequences of the primers used in this study are described below

β-actin: 5'-GAGCACAGAGCCTCGCCTTT-3' and 5'-ATCCTTCTGACCCATGCCCA-3'. SHANK2: 5'-CGGGTAATCCTCCCAAATCA-3' and 5'-CTTTATCCCGGCGTTTCATC-3'.

### Lentiviral production and infection

The lentivirus packaging vectors used were psPAX2 (Addgene, Cambridge, MA, USA) and pMD2.G (Addgene). Generation of lentivirus in HEK-293T cells and transfection of lentiviral constructs into recipient cell lines were performed according to the manufacturer’s instructions (Thermo Fisher Scientific, Carlsbad, CA, USA). Transfection reagent polyethylenimine (PEI) was purchased from Sigma-Aldrich.

### Transwell migration and invasion assays

Migration and invasion were evaluated by plating 2.5 × 10^4^ cells in the upper chambers of 8.0 μm pore size reduced growth factor Matrigel chambers or control non-coated chambers (BD Biosciences) in 0.5% FBS/DMEM. Cells were allowed to invade for 24 hr towards DMEM/10% fixed with ice-cold methanol, and stained with 0.5% crystal violet. Two chambers per condition in three independent experiments were imaged at 5x and four fields per chamber were counted and analyzed.

### Immunofluorescence staining

The cells were washed three times with PBS and were fixed for 15 min at room temperature with 4% (vol/vol) paraformaldehyde and permeabilized with 0.2% Triton X-100 for 20 min on ice. Following permeabilization, nonspecific binding in the cells was blocked by incubation for 30 min at room temperature with 5% BSA in PBS and cells were incubated for 2 hr with specific primary antibodies (identified above, antibodies indicated in figures). After three washes with PBS, the cells were incubated for another 1 hr with secondary antibodies Alexa Fluor 488–conjugated anti–mouse IgG (A21202), Alexa Fluor 488–conjugated anti–rabbit IgG (A21206) or Alexa Fluor 555–conjugated anti–mouse IgG (A31570) (all from Invitrogen). Nuclei were counterstained with DAPI (4, 6-diamidino- 2-phenylindole; Sigma-Aldrich). All images were collected with a confocal microscope (Zeiss LSM 780).

### Glutathione S-transferase pull-down assay

Briefly, GST, GST-PRMT7 protein expressions were induced by adding 0.1 mmol/L IPTG at 25°C for 8 hr with shaking, and then purified on glutathione-Sepharose4B according to the manufacturer's instructions (GE Healthcare).

### Affinity purification of Flag-tagged proteins

HEK293T cells were transfected with pWPXLD-3xflag-PRMT7 plasmid, using the PEI reagent according to the manufacturer’s instructions. After transfection for 48 hr, cells were harvested and lysed in the buffer A containing protease inhibitor cocktail tablet (Roche). Total cell extracts were incubated with anti-Flag affinity gel (Biotool, Kirchberg, Switzerland) for 3 hr at 4°C, and the immunoprecipitates were washed 3 times with 13 Tris-buffered saline buffer [50 mM Tris-HCl (pH 7.4) and 150 mM NaCl]. Finally, the bound proteins were eluted with 3xflag peptide (ApexBio, Houston, TX, USA) for 1 hr at 4°C.

### In vitro SHANK2 methylation assay

HA-SHANK2 (5 μg) was incubated with GST-PRMT7 in the presence of S-adenosyl-methionine (SAM; 15 Ci/mmoL; PerkinElmer, Waltham, MA, USA) at 30°C for 1 hr. The reaction was stopped by adding loading buffer followed by SDS PAGE.

### Structure analysis

The SHANK2 (NP_036441.2) structure was homology modelled via SWISS-MODEL web server based on the template of PDB ID 5G4X with the identity of 69%. The wild type SHANK2 model and the mutant one (Arg240Lys) were solvated in ~32,000 TIP3P water molecules with 150 mM NaCl in a 116 × 116 × 80 Å box. Both systems were built and pre-equilibrated with the CHARMM program using the CHARMM36 force field. The systems were equilibrated for 25ns using the NAMD2.12 program package under the periodic orthorhombic boundary conditions applied in all directions with the time step of 2 fs. The NPT ensemble was used for both simulations with pressure set to one atm and temperature to 310.15 K. Long-range electrostatic interactions were treated by the particle mesh Ewald (PME) algorithm. Non-bonded interactions were switched off at 10–12 Å.

### MS analysis

Flag-PRMT7 protein was purified from Flag-PRMT7- MDA-MB-231 cells and was then resolved by 10% SDS-PAGE. After Coomassie brilliant blue staining, the band corresponding to Flag-PRMT7 was excised for liquid chromatography-tandem mass spectrometry (LC–MS/MS) analysis performed in the Institute of Biophysics (Chinese Academy of Sciences, Beijing, China).

HA-SHANK2 protein was purified from HA-SHANK2-MDA-MB-231 cells and was then resolved by 10% SDS-PAGE. After Coomassie brilliant blue staining, the band corresponding to HA-SHANK2 was excised for liquid chromatography-tandem mass spectrometry (LC–MS/MS) analysis performed in the Institute of Biophysics (Chinese Academy of Sciences, Beijing, China).

### Breast cancer specimen collection

Human breast tumour specimens were obtained from the Second Hospital of Jilin University, China. All the breast cancer tissue samples were collected from 27 patients enrolled on pathology department of the Second Hospital of Jilin University. All the samples were diagnosed by the pathology department of the Second Hospital of Jilin University to determine the stage and subtype of the breast tumour (Supplementary file 1 and Supplementary file 2). This experiment is an immunohistochemical study, no informed consent was needed due to the use of post-diagnostic left-over material. Ethical approval was obtained from the Ethics Review Committee of the Second Hospital of Jilin University (2019–107).

### TCGA data analysis

The Cancer Genome Atlas (TCGA) Breast cancer (BRCA) dataset was retrieved from http://cancergenome.nih.gov. Samples with clinical information and mRNA expression data were selected (1075 samples data) to evaluate the correlation between PRMT7 and the pathological stage of breast cancer patients.

### Histologic evaluation and immunohistochemical staining

The IHC staining was performed using a VECTASTAIN ABC kit according to the manufacturer’s instructions. Sections of patients with breast cancer were stained with antibodies against PRMT7, p-FAK or p-cortactin. The following proportion scores were assigned: 0, 1, 2, 3 and 4 if 0%, 0–10%, 11–50%, 51–75%, and 76–100% of the tumour cells exhibited positive staining, respectively. Also, the staining intensity was rated on a scale of 0 to 3: 0, negative; 1, weak; 2, moderate; and 3, strong. The proportion and intensity scores were then multiplied to obtain a total score.

### Animal studies

MDA-MB-231-shSHANK2-Vector, MDA-MB-231-shSHANK2 with SHANK2 WT or SHANK2 R240K (2 × 10^6^) cells were injected into tail-vein of 5-week-old female BALB/c nude mice. Following tumour cell injection, the mice were randomized (n = 5 mice per group) according to the following groups: 1 100 μL of a vehicle control (oral, daily; 2) 75 mg/kg GSK2256098 in 100 μL of vehicle (oral, daily); Therapy was initiated 10–14 days after tumour injection. Six weeks later, the mice were sacrificed and lungs fixed in formalin before embedded in paraffin using the routine procedure. Hematoxylin and eosin (H and E) staining was performed on sections from paraffin-embedded tissues. All the mice were housed in specific-pathogen free (SPF) conditions. All animal works were conducted in accordance with the IACUC guidelines and with the protocol approved by the IACUC of Northeast Normal University, reference assurance number AP2013011.

### Statistical analysis

Statistical analyses were performed using GraphPad Prism five software. Statistical parameters and methods are reported in the Figures and the Figure Legends. Unless specified, comparisons between groups were made by unpaired two-tailed Student’s *t-*test. A value of p<0.05 was considered statistically significant. For the correlation between PRMT7 expression and stage of breast cancer patients, a chi2 test was used, and the differences were considered as significance at p<0.05. A simultaneous comparison of more than two groups was conducted using one-way ANOVA (SPSS statistical package, version 12; SPSS Inc). Values of p<0.05 were considered statistically significant.

## Data Availability

PDB accession number for SHANK2 structure analyse is pdb5G4X. Analysis of SHANK2 gene expression in human tissues using the Human Protein Atlas data. The following previously published dataset was used: LiljaJZacharchenkoTGeorgiadouMJacquemetGFranceschiNPeuhuEHamidiHPouwelsJMartensVNiaFHBeifussMBoeckersTKreienkampHJBarsukovILIvaskaJ2019The crystal structure of the SHANK3 N-terminusRCSB Protein Data Bank5G4X

## Additional files

Supplementary file 1. Clinical breast cancer adjacent tissues.

Supplementary file 2. Clinical breast cancer tissues.

Transparent reporting form

## Appendix 1

### Key resources table

**Appendix 1—key resources table:**

Reagent type (species) or resource	Designation	Source or reference	Identifiers	Additional information
Antibody	Anti- N-cadherin (Mouse monoclonal)	BD Biosciences	Cat# 561553, RRID:AB_10713831	WB (1:1000)
Antibody	Anti- fibronectin (Mouse monoclonal)	BD Biosciences	Cat# 610070, RRID:AB_2105706	WB (1:1000)
Antibody	Anti-β-catenin (Mouse monoclonal)	BD Biosciences	Cat# 610154	WB (1:1000)
Antibody	Anti- EEA1 (Mouse monoclonal)	BD Biosciences	Cat# 610456, RRID:AB_397829	IF (1:100)
Antibody	Anti- Rab5 (Mouse polyclonal)	BD Biosciences	Cat# 610724, RRID:AB_398047	IF (1:100)
Antibody	Anti-β-actin (Mouse monoclonal)	Sigma-Aldrich	Cat# A5228, RRID:AB_262054	WB (1:5000)
Antibody	Anti- HA (Mouse monoclonal)	Sigma-Aldrich	Cat# H9658, RRID:AB_260092	WB (1:1000) IP (4 μg)
Antibody	Anti- MMP2 (Rabbit polyclonal)	GeneTex	Cat# GTX-104577 RRID:AB_1950932	WB (1:1000)
Antibody	Anti-MMP9 (Rabbit polyclonal)	GeneTex	Cat# 40086	WB (1:1000)
Antibody	Anti- p-cortactin (Rabbit polyclonal)	Bioworld	Cat# BS4778, RRID:AB_1663129	IHC (1:100)
Antibody	Anti- p-cortactin (Rabbit polyclonal)	Abcam	Cat# ab47768, RRID:AB_869231	WB (1:1000)
Antibody	mono methyl Arginine (Mouse monoclonal)	Abcam	Cat# ab415, RRID:AB_304323	WB (1:500)
Antibody	asymmetric dimethyl Arginine(Mouse monoclonal)	Abcam	Cat# ab412, RRID:AB_304292	WB (1:500)
Antibody	Dyn2 (Rabbit polyclonal)	Abcam	Cat# ab3457, RRID:AB_2093679	WB (1:1000) IF (1:100)
Antibody	Flag (Mouse monoclonal)	Abmart	Cat# M20008, RRID:AB_2713960	WB (1:1000)
Antibody	p-FAK (Rabbit polyclonal)	Invitrogen	Cat# 700255, RRID:AB_2532307	IHC (1:100) IP (4 μg)
Antibody	PRMT7(Mouse monoclonal)	santa cruz	Cat# sc-376077, RRID:AB_10990266	IHC (1:200)
Antibody	PRMT7 (Rabbit monoclonal)	Cell Signaling Technology	Cat# 14762, RRID:AB_2798599	WB (1:1000) IP (4 μg) IF (1:100)
Antibody	SHANK2 (Rabbit polyclonal)	Cell Signaling Technology	Cat# 12218, RRID:AB_2797848	WB (1:500) IP (4 μg) IF (1:100)
Antibody	p-FAK(Rabbit monoclonal)	Cell Signaling Technology	Cat# 8556, RRID:AB_10891442	WB (1:1000)
Antibody	FAK (Rabbit polyclonal)	Cell Signaling Technology	Cat# 3285, RRID:AB_2269034	WB (1:1000) IF (1:100)
Antibody	p-talin(Rabbit monoclonal)	Cell Signaling Technology	Cat# 13589, RRID:AB_2798267	WB (1:1000)
Antibody	talin(Rabbit monoclonal)	Cell Signaling Technology	Cat# 4021, RRID:AB_2204018	WB (1:1000) IF (1:100)
Antibody	ZO-1(Rabbit polyclonal)	Cell Signaling Technology	Cat# 5406, RRID:AB_1904187	WB (1:1000)
Antibody	symmetric dimethyl Arginine(Rabbit polyclonal)	Millipore	Cat# 07–412, RRID:AB_11212396	WB (1:500)
Antibody	PRMT5(Rabbit polyclonal)	Millipore	Cat# 07–405, RRID:AB_310589	WB (1:1000)
Antibody	cortactin(Mouse monoclonal)	Millipore	Cat# 16–228, RRID:AB_441969	WB (1:1000) IF (1:100)
Sequenced-based reagent	Interference in the primer:PRMT7#1	Addgene		GGAACAAGCTATTTCCCATCC
Sequenced-based reagent	Interference in the primer:PRMT7#2	Addgene		GGATGCAGTGTGTGTACTTCC
Sequenced-based reagent	Interference in the primer:SHANK2#1	Addgene		GGAGTTAGTCAAAGCACAAAG
Sequenced-based reagent	Interference in the primer:SHANK2#2	Addgene		GCTTGGAGCAAGAGAGAATTT
Sequenced-based reagent	Interference in the primer:shEEA1#1	Addgene		GCGGAGTTTAAGCAGCTACAA
Sequenced-based reagent	PCR Primer: β-actin forward:	Addgene	PCR Primers	GAGCACAGAGCCTCGCCTTT
Sequenced-based reagent	PCR Primer: β-actin reverse:	Addgene	PCR Primers	ATCCTTCTGACCCATGCCCA
Sequenced-based reagent	PCR Primer: SHANK2 forward:	Addgene	PCR Primers	CGGGTAATCCTCCCAAA
Sequenced-based reagent	PCR Primer: SHANK2 reverse:	Addgene	PCR Primers	CTTTATCCCGGCGTTTCATC
Recombinant DNA reagent	Flag-cortactin (plasmid)	The lab of Dr. Alpha S. Yap.This paper		
Recombinant DNA reagent	HA-SHANK2 (plasmid)	The lab of Dr. Min Goo Lee.This paper		
Recombinant DNA reagent	pcDNA3-HA-SHANK2 (plasmid)	Addgene		
Recombinant DNA reagent	pWPXLD-SHANK2 (plasmid)	Addgene		
Recombinant DNA reagent	pWPXLD-Flag-PRMT7 (plasmid)	Addgene		
Recombinant DNA reagent	pWPXLD-PRMT7 (plasmid)	Addgene		
Recombinant DNA reagent	pWPXLD-Flag-PRMT5 (plasmid)	Addgene		
Recombinant DNA reagent	pWPXLD-PRMT5 (plasmid)	Addgene		
Chemical compound, drug	Dynasore	Selleck	Cat# S8047	
Chemical compound, drug	GSK591	Selleck	Cat# S8111	
Chemical compound, drug	GSK2256098	Selleck	Cat# S5823	
Chemical compound, drug	EGF	Sigma-Aldrich	Cat# E9644	
Chemical compound, drug	hydrocortisone	Sangon	Cat# A610506	
Chemical compound, drug	cholera toxin	Sigma-Aldrich	Cat# C8180	
Chemical compound, drug	insulin	Gibco, Grand Island, NY, USA	Cat# 12585–014	
Chemical compound, drug	hFGF basic	R and D Systems, Minneapolis, MN, USA	Cat# P09038	
Strain, strain background *Mus musculus*	BALB/c nude (CAnN.Cg-*Foxn1^nu^*/Crl)	Charles River Labs	Cat#CRL:194,RRID:IMSR_CRL:194	
Cell line (*Homo-sapiens*)	MCF10A (human; female)	American Type Culture Collection	Cat# CRL-10317, RRID:CVCL_0598	
Cell line (*Homo-sapiens*)	MCF7 (human; female)	American Type Culture Collection	Cat# HTB-22, RRID:CVCL_0031	
Cell line (*Homo-sapiens*)	T47D (human; female)	American Type Culture Collection	Cat# HTB-133, RRID:CVCL_0553	
Cell line (*Homo-sapiens*)	BT474(human; female)	American Type Culture Collection	Cat# HTB-20, RRID:CVCL_0179	
Cell line (*Homo-sapiens*)	MDA-MB-231(human; female)	American Type Culture Collection	Cat# HTB-26, RRID:CVCL_0062	
Cell line (*Homo-sapiens*)	BT549(human; female)	American Type Culture Collection	Cat# HTB-122, RRID:CVCL_1092	
Cell line (*Homo-sapiens*)	HEK293T (human; fetus)	American Type Culture Collection	Cat# CRL-3216, RRID:CVCL_0063	
Software, algorithm	ImageJ	Wayne Rasband, National Institutes of Health	RRID:SCR_003070	
Software, algorithm	GraphPad Prism 8	GraphPad Software	Version 8.3 RRID:SCR_002798	
